# Effect of Dihuang Yinzi on Inflammatory Response in Cerebral Ischemia-Reperfusion Model Rats by Regulating Gut Microbiota

**DOI:** 10.1155/2022/3768880

**Published:** 2022-08-17

**Authors:** Xinyu Wang, Lei Ye, Wanru Sun, Liya Li, Chaoyun Wang, Xiaoyan Xu, Zhaohai Pan, Jianwei Gong

**Affiliations:** Binzhou Medical University, Laishan District, Yantai, 264003 Shandong, China

## Abstract

Dihuang Yinzi, as a classical Chinese medicine prescription, plays an important role for the treatment of ischemic stroke. Gut microbiota play a functional role for the expression of proinflammatory cytokines and anti-inflammatory cytokines, which further affect central nervous system and change brain function. Our research confirmed that Dihuang Yinzi can exert brain protection by inhibiting inflammatory reaction. Dihuang Yinzi can significantly decrease the contents of interleukin-6 (IL-6), tumor necrosis factor-*α* (TNF-*α*), and interleukin-17 (IL-17) in brain, serum, and colon tissues and increase the contents of transforming growth factor-*β* (TGF-*β*) and interleukin-10 (IL-10) in cerebral ischemia-reperfusion model rats. The results of 16s rRNA high-throughput sequencing showed that Dihuang Yinzi had a significant effect on microbiome in rats. The firmicutes, bacteroidetes, and proteobacteria were dominant in Dihuang Yinzi group. The content of firmicutes increased with the increase of dosage of Dihuang Yinzi. Especially, the content of actinomycetes in the high-dose group was higher than other groups. At the genus level, the number of bacteroides in the antibiotic groups was significantly higher than that in the other treatment groups. The results suggest that Dihuang Yinzi may play important roles in treatment of ischemic stroke by regulating the gut microbiota and the inflammatory reaction in the colon tissues, serum, and brain of the model rats, to verify the scientific nature of this prescription in relieving brain inflammatory reaction and brain injury by this way and to reveal the brain-gut related mechanism of Dihuang Yinzi in treating ischemic stroke.

## 1. Introduction

Ischemic stroke, the most common type of stroke, occurs when a blood vessel in the neck or brain is blocked [1]. Ischemic stroke is a common disease among middle-aged and elderly people with high incidence, disability, and recurrence rate, which seriously affects the physical and mental health and quality of life of human beings. The reports indicated, in the United States, that more than 795,000 individuals have a stroke each year [2]. The increasing researches suggested that the brain and gastrointestinal tract were involved in complex bidirectional regulation through the neuro-immune-endocrine-gut microbiota [3, 4]. According to the survey of the intensive care unit (ICU) patients, most patients, in the early stage of stroke, are in a state of high stress, which can lead to a strong systemic inflammatory response, leading to intestinal dynamic disorder, imbalance of flora, ischemia, excessive growth of cytokines, lack of cytokines, and excessive apoptosis of intestinal mucosal epithelial cells, resulting in intestinal mucosal barrier injury. Therefore, we speculate that regulating intestinal function and intestinal microbiota can treat stroke patients to a certain extent [5].

Dihuang Yinzi is based on the theory of traditional Chinese medicine (TCM) and has the function of nourishing kidney yin and nourishing essence [6]. Studies have found that Dihuang Yinzi has good effect in antioxidative damage, inhibiting nerve cell apoptosis and promoting the formation of new blood vessels in the ischemic area of cerebral tissue in the cerebral infarction rats [7]. Gut microbes act on the immune system, make proinflammatory and anti-inflammatory cytokines change, affect the central nervous system, and change brain function. Translational studies manifest that some of the bacteria may have effects on stress responses and cognitive function, shedding new light on manipulating the gut microbiome with antibiotics to alter brain function [8]. Therefore, we speculated Dihuang Yinzi treats ischemic stroke by improving intestinal microecology and regulating the inflammatory state in vivo.

In this study, we systematically examined the changes of intestinal flora before and after rat modeling and the regulatory effects of each drug on intestinal flora by using microbiome. The mechanism of brain-intestine connection in the treatment of ischemic stroke with Dihuang Yinzi was revealed. It provides the basis for the rational use of Dihuang Yinzi and is also of great significance to improve the evolution of gastrointestinal syndrome in the course of stroke.

## 2. Materials and Method

### 2.1. Animals

60 healthy male SD rats weighing 250-300 g were purchased from Pengyue. The animal license no. SCXK (lu) was 20190003. 42 rats were divided into 7 groups, including sham operation group; model 1 group; model group; high-, intermediate-, and low-dose groups of Dihuang Yinzi; and antibiotic group (amoxicillin/clavulanic acid) (Figure 1). The rat model of cerebral ischemia-reperfusion was established by clipping the common carotid arteries. Intragastric administration was started on the second day after modeling, once a day for 7 consecutive days. The experiments were approved by the Binzhou Medical University Animal Care and Use Committee.

### 2.2. Model Building Method

The rats were anesthetized and fixed on the supine position. The anterior cervical skin was cut open, the bilateral common carotid artery was separated along the left and right trachea, and the bilateral common carotid artery was closed with noninvasive artery clip for 30 min, resulting in acute cerebral ischemia. Loosen the artery clamp after 30 min reperfusion, reoccupy after 30 min noninvasive arterial clip on both sides of common carotid arteries 30 min, and the mold is finished after loosening and stitching. After separation and in the process of bilateral common carotid artery clamping and loosening, gauze soaked in warm saline was used to cover the incision surface to keep the tissue moist. The operation method of sham-operated group was the same as that of the model group, but the common carotid artery on both sides was not clipped.

### 2.3. Gene Sequencing

16S rRNA sequencing and conducted were performed as previously described [9]. In brief, the QIAamp Fast DNA Stool Mini Kit (Qiagen, California, USA) was selected to extract the bacterial genomic DNA. The 16SrRNA V3-V4 region was used to amplify by using PCR and then sequenced with MiSeq platform.

### 2.4. The Levels of Inflammatory Cytokines in Rats Were Detected

Reagent of IL-6 (batch number: E20191204-30219a), TNF-*α* (batch number: e20191201-31063a), IL-17 (batch number: e20191202-30201a), TGF-*β* (batch number: e20191206-31072a), and IL-10 (batch number: e20191203-30194a) were purchased from Shanghai Enzyme-Linked Biotechnology Co., Ltd. Blood was collected from the rat heart, centrifuged at 4°C at 3000 r/min for 15 min, and serum was collected and stored at -80°C. The cortical tissue and colon tissue of the rat separately were removed from the ice and diluted after homogenization. The contents of proinflammatory factors IL-6, TNF-*α*, and IL-17and anti-inflammatory factors TGF- and IL-10 in the cerebral cortex and serum of rats were detected by ELISA.

### 2.5. Bioinformatic Analysis

Quantitative Insights Into Microbial Ecology was used to process the 16S rRNA sequencing data [10]. Sequencing reads was filtered, and feature table was constructed by DADA2 software. Then, vsearch plugin was used to cluster sequences into OTUs at 97% identity [11]. MAFFT [12] was selected to align the sequences, and a phylogenetic tree was generated with FastTree plugin. Q2-diversity was used to conduct alpha and beta diversity analyses. The metagenomes of gut microbiome were processed from 16S rRNA sequences using PICRUSt as described before [13]. The raw sequence data has been submitted to the NCBI Short Read Archive with accession number PRJNA628126.

### 2.6. Statistical Analysis

LEfSe analysis was applied to distinguish taxa or pathways in different group [14]. Fisher's exact test [15] and Kruskal-Wallis test [16] also were adopted to analyze the data. SPSS 23.0 statistical software was used for statistical methods, and *t* test was used for measurement data.

## 3. Results

### 3.1. Effect of Dihuang Yinzi on the Content of Inflammatory Factors in Cerebral Cortex, Serum, and Colonic Tissues of Rat

Combined with previous findingss, our resultsindicated that, stroke model group compared with sham group, the contents of IL-6, TNF-*α*, and IL-17 in cerebral cortex, serum, and colonic tissues were significantly increased (*P* < 0.05), and contents of TGF-*β* and IL-10 obviously were decreased (*P* < 0.05), demonstrating severe inflammatory reaction occurred in rats. Meanwhile, Dihuang Yinzi can significantly reduce content of IL-6, TNF-*α*, and IL-17 (*P* < 0.05) and increase the contents of TGF-*β* and IL-10 (*P* < 0.05), which is verified that this prescription can control the inflammatory reaction. Dihuang Yinzi can reduce the damage of brain tissue and play a protective role in brain by correcting the imbalance between proinflammatory factors and anti-inflammatory factors in vivo after cerebral ischemia (Table 1–6).

### 3.2. Faecal Bacterial Diversity in Rats with Ischemia Apoplexy

*α*-Diversity can effectively detect taxa richness and evenness, and *β*-diversity compares the similarity or difference in communities between sample. *α*-Diversity indices were employed to compare the richness estimators (Chao1 and Ace) and diversity index (Figure 2). We found that the gut microbiome of rehmanniae group was markedly more diverse compared to antibiotic group. However, it has no significant changes at the three rehmanniae groups (D, E, and F groups). To further explore the effect of Dihuang Yinzi on microbiomes analysis, *β*-diversity (PCoA) was adopted to reveal microbiome community structures similarities (Figure 3), which showed that the microbiota of antibiotic group differed substantially from other individuals. Similar to alpha diversity, it displays the similarity of microbiome community structures in three rehmanniae groups.

### 3.3. Bacteria Differentially Abundant in Different Treatment Group

Community structure were compared, indicating that firmicutes, bacteroidetes, and proteobacteria were the most predominant phyla, and the content of firmicutes keep increasing with improvement of rehmanniae dose (Figure 4(a)). Especially, the content of actinobacteria in the high-dose group was the highest than other groups. At the genus level, bacteroides in the high-dose group was also higher than other treatment groups (Figure 4(b)). In all groups, Lactobacillus in the high-dose group was evidently lower than other groups (Figure 4).

LEfSe analysis was conducted to the faecal microbiota composition among 7 treatment group to identify differentially abundant taxa.  Figure 5(a) shows that the taxa differed most between different communities. 43 discriminative features were found by LEfSe analysis (LDA score > 4) (Figure 5(b)). 10, 5, and 5 bacteria were significantly more abundant in sham-operated group, model 1 group, and model group, separately. The allobaculum, christensenellaceae, and ruminococcaceae were enriched in the high-dose group. Ruminococcaceae and coprostanoligenes were more abundant in the low-dose group. Ten bacteria including bacteroides, bacteroidaceae, enterobacteriaceae, shigella, and blautia were enriched in antibiotics groups (Figure 5).

### 3.4. Microbial Functional Dysbiosis in Samples

PICRUSt was used to analyze the potential function of the gut microbiota. The results showed that the proportion of digestive system in the microbiome of the sham group was higher than that of the model group. Energy metabolism was also higher in antibiotics groups. Additionally, global and overview maps was significantly increased in the antibiotics groups (Figure 6).

## 4. Discussion

Gut microbiota is closely correlated with stroke, and the research has indicated that the microbiota is altered after experimental stroke in young rats [17–19]. Here, Dihuang Yinzi on the gut microbiota has been investigated. The results revealed that Dihuang Yinzi had a protective effect against ischemia apoplexy, decreased the content of proinflammatory factors, and increased the content anti-inflammatory factors. Additionally, Dihuang Yinzi was found to modulate the gut microbiota, enhancing more beneficial microorganisms growth, while suppressing the growth of potential pathogens.

The contents of IL-6, TNF-*α*, and IL-17 and anti-inflammatory factors TGF-*β* and IL-10 in cerebral, cortex serum, and colon tissue were determined, indicating that Dihuang Yinzi can significantly reduce the levels of IL-6, TNF-*α*, and IL-17 and improve the contents of TGF-*β* and IL-10. Studies indicated that NK cells, B lymphocytes, and TNF-*α*, TGF-*β*, CRP, IL-4, IL-6, and IL-10 are altered after stroke [20–22]. Dihuang Yinzi may act as anti-inflammatory protection after stroke in cerebral, cortical serum, and colon tissue, such as TGF-*β* and IL-10, decrease content of proinflammatory factor including IL-6, TNF-*α*, and IL-17 and may play protective roles on stroke.

Recently, increasing researchers set out to study the effect of gut microbiota on stroke and to explore the reconfiguration of microbial community in experimental models after stroke of humans and rats. Tascilar et al. found that bacterial translocated to extraintestinal structures in a mouse MCAO [23]. Caso et al. reported bacterial translocation to different body parts in stress before MCAO in the experiment of rats [24]. Winek et al. indicated that several bacteria were abrupt disappearance after stroke after acute brain injury [25]. We discovered that the gut microbiome of model group was markedly more diverse compared to sham-operated group. Compared with model group, the microbiome of the sham group had a higher proportion of the digestive system. After a stroke, the function associated with digestion is reduced, and presumably, microorganisms related with digestion were decreased. Results found that the content of actinobacteria in the high-dose group was higher than other group. Lactobacillus in the high-dose group was evidently lower than other group. Especially, the content of prevotellaceae in Dihuang Yinzi groups was lower than that of the model group. The study by Yamashiro et al. showed that stroke patients had significantly higher rumen Lactobacillus bacteria counts compared with controls [26]. Therefore, we suspect that Dihuang Yinzi inhibits the growth of Lactobacillus.

A high-risk group for stroke had an enrichment of opportunistic pathogens and lactate-producing bacteria, but a decrease in butyrate-producing bacteria, compared with a low-risk group for stroke, one report showed [27], which explain the reason for the increase of allobaculum, christensenellaceae, and ruminococcaceae et al., in Dihuang Yinzi groups. The consumption of a diet containing rehmanniae is conducive to the accumulation of more beneficial microorganisms while inhibiting the growth of potential pathogens [28]. Furthermore, we also analyzed the effect of antibiotics on the intestinal bacteria. Results showed that antibiotics significantly changed microbiota. Compared with other groups, the species and number of microorganisms were significantly decreased. Researches indicated that antibiotics which altered the gut microbiota reduced neurological impairment and the cerebral infarct volume [29].

In conclusion, our results reveal that Dihuang Yinzi can significantly reduce content of IL-6, TNF-*α*, and IL-17, improve the content of TGF-*β* and IL-10, and modulate the gut microbiota, promoting a decrease of the ratio of lactobacillus and increasing the relative abundance of allobaculum, christensenellaceae, and ruminococcaceae. Thereby, it provides a new approach against ischemia apoplexy.

## Figures and Tables

**Figure 1:** An overview of the study design and timeline. One mouse from each cage was treated according to experiment condition (*N* = 42, 6 mice per group).

**Figure 2:** Diversity estimation of the 16S rRNA gene. (a) ACE indice; (b) Chao indice; (c) Shannon indice.

**Figure 3:** PCoA based on unweighted UniFrac matrix showed that the overall faecal microbiota composition was different in different group.

**Figure 4:** Relative abundances of the gut microbiota at phylum level (a) and genus level (b).

**Figure 5:** Taxonomic differences in 7 group by LEfSe and LDA. (a) LEfSe results for the bacterial communities. (b) Cladogram using the LDA model results for the bacterial hierarchy.

**Figure 6:** Functional analyses of predicted metagenomes. (a) Differentially abundant KEGG pathways across A and C groups. (b) Differentially abundant KEGG pathways across C and G groups.

**Table 1:** Effects of Dihuang Yinzi on levels of proinflammatory factors Il-6, TNF-*α*, and Il-17 in the cerebral cortex of rats.

Group	IL-6 (pg/g)	TNF-*α* (pg/g)	IL-17 (pg/g)
Sham-operated group	733.74 ± 9.26	1837.90 ± 21.00	93.57 ± 15.11
Model group	1915.10 ± 41.80^##^	3887.68 ± 61.57^##^	527.04 ± 37.52^##^
Low-dose group	1713.59 ± 26.52^∗^	3242.96 ± 43.84^∗∗^	430.16 ± 21.67^∗∗^
Intermediate-dose group	1396.17 ± 15.95^∗∗^	2749.47 ± 29.54^∗∗^	320.34 ± 13.35^∗∗^
High-dose group	1187.95 ± 26.22^∗∗^	2347.12 ± 24.70^∗∗^	280.35 ± 11.54^∗∗^
Antibiotics group	1132.88 ± 24.75^∗∗^	2157.77 ± 28.47^∗∗^	181.59 ± 6.13^∗∗^

^##^ *P* < 0.01 compared with sham-operated group; ^∗^*P* < 0.05, ^∗∗^*P* < 0.01 compared with model group.

**Table 2:** Effect of Dihuangyinzi on the contents of anti-inflammatory factors TGF-*β* and IL-10 in rat cerebral cortex.

Group	TGF-*β* (pg/g)	IL-10 (pg/g)
Sham-operated group	2637.56 ± 42.76	934.68 ± 24.68
Model group	646.28 ± 30.35^##^	543.32 ± 39.92^##^
Low-dose group	1105.80 ± 24.74^∗∗^	629.47 ± 23.56^∗∗^
Intermediate-dose group	1438.53 ± 37.76^∗∗^	677.57 ± 19.33^∗∗^
High-dose group	1895.97 ± 43.35^∗∗^	769.12 ± 32.32^∗∗^
Antibiotics group	2137.29 ± 32.09^∗∗^	846.06 ± 31.02^∗∗^

^##^ *P* < 0.01 compared with sham-operated group; ^∗∗^*P* < 0.01 compared with model group.

**Table 3:** Effects of Dihuang Yinzi on serum levels of proinflammatory factors Il-6, TNF-*α*, and Il-17 in rats.

Group	IL-6 (pg/ml)	TNF-*α* (pg/ml)	IL-17 (pg/ml)
Sham-operated group	88.42 ± 2.22	153.33 ± 2.38	10.53 ± 0.64
Model group	221.05 ± 7.86^##^	414.32 ± 10.91^##^	58.57 ± 2.47^##^
Low-dose group	186.60 ± 4.23^∗∗^	351.01 ± 6.40^∗∗^	46.21 ± 2.56^∗∗^
Intermediate-dose group	171.70 ± 2.53^∗∗^	300.87 ± 8.09^∗∗^	36.55 ± 1.10^∗∗^
High-dose group	140.46 ± 2.85^∗∗^	262.73 ± 5.53^∗∗^	31.71 ± 1.91^∗∗^
Antibiotics group	119.64 ± 4.89^∗∗^	218.36 ± 11.66^∗∗^	19.70 ± 0.67^∗∗^

^##^ *P* < 0.01 compared with sham-operated group; ^∗∗^*P* < 0.01 compared with model group.

**Table 4:** Effect of Dihuang Yinzi on serum levels of anti-inflammatory factors TGF-*β* and IL-10 in rats.

Group	TGF-*β* (pg/ml)	IL-10 (pg/ml)
Sham-operated group	282.32 ± 4.25	93.52 ± 1.81
Model group	87.48 ± 2.29^##^	52.19 ± 3.22^##^
Low-dose group	120.34 ± 2.17^∗∗^	60.94 ± 2.69^∗∗^
Intermediate-dose group	155.97 ± 7.42^∗∗^	73.80 ± 1.22^∗∗^
High-dose group	194.43 ± 5.07^∗∗^	81.13 ± 3.26^∗∗^
Antibiotics group	242.30 ± 7.51^∗∗^	90.77 ± 4.30^∗∗^

^##^ *P* < 0.01 compared with sham-operated group; ^∗∗^*P* < 0.01 compared with model group.

**Table 5:** Effects of Dihuang Yinzi decoction on the contents of proinflammatory factors Il-6, TNF-*α*, and Il-17 in colon tissues of rats.

Group	IL-6 (pg/g)	TNF-*α* (pg/g)	IL-17 (pg/g)
Sham-operated group	753.36 ± 33.90	1536.40 ± 26.25	156.88 ± 1.87
Model group	1914.23 ± 23.49^##^	3317.93 ± 52.33^##^	585.88 ± 13.06^##^
Low-dose group	1594.68 ± 27.84^∗∗^	3203.75 ± 48.85^∗^	444.11 ± 15.23^∗∗^
Intermediate-dose group	1369.23 ± 38.96^∗∗^	2759.59 ± 54.46^∗∗^	344.76 ± 9.04^∗∗^
High-dose group	1233.13 ± 16.20^∗∗^	2356.35 ± 47.34^∗∗^	324.67 ± 10.86^∗∗^
Antibiotics group	847.22 ± 21.69^∗∗^	2241.24 ± 9.13^∗∗^	247.39 ± 3.98^∗∗^

^##^ *P* < 0.01 compared with sham-operated group; ^∗^*P* < 0.05, ^∗∗^*P* < 0.01 compared with model group.

**Table 6:** Effect of Dihuang Yinzi on contents of anti-inflammatory factors TGF-*β* and Il-10 in colon tissues of rats.

Group	TGF-*β* (pg/g)	IL-10 (pg/g)
Sham-operated group	2800.04 ± 45.29	910.33 ± 18.25
Model group	946.28 ± 27.49^##^	421.83 ± 7.30^##^
Low-dose group	1255.37 ± 51.88^∗∗^	571.00 ± 11.78^∗∗^
Intermediate-dose group	1494.92 ± 62.90^∗∗^	642.28 ± 15.82^∗∗^
High-dose group	1828.07 ± 38.31^∗∗^	727.52 ± 6.92^∗∗^
Antibiotics group	2277.89 ± 15.58^∗∗^	772.17 ± 13.46^∗∗^

^##^ *P* < 0.01 compared with sham-operated group; ^∗∗^*P* < 0.01 compared with model group.

## Data Availability

Data to support the findings of this study is available on reasonable request from the corresponding author.

## References

[1] Mozaffarian D., Benjamin E. J., Go A. S. (2016). Heart disease and stroke statistics-2016 update: a report from the American Heart Association. *Circulation*.

[2] Randolph S. A. (2016). Ischemic stroke. *Workplace Health & Safety*.

[3] Mayer E. A., Tillisch K., Gupta A. (2015). Gut/brain axis and the microbiota. *The Journal of Clinical Investigation*.

[4] Tache Y., Larauche M., Yuan P. Q., Million M. (2018). Brain and gut CRF signaling: biological actions and role in the gastrointestinal tract. *Current Molecular Pharmacology*.

[5] Galland L. (2014). The gut microbiome and the brain. *Journal of Medicinal Food*.

[6] Yuan H., Yang M., Han X., Ni X. (2018). The therapeutic effect of the Chinese herbal medicine, rehmanniae Radix preparata, in attention deficit hyperactivity disorder via reversal of structural abnormalities in the cortex. *Cortex*.

[7] Liu C., Ma R., Wang L. (2017). *Rehmanniae Radix* in osteoporosis: a review of traditional Chinese medicinal uses, phytochemistry, pharmacokinetics and pharmacology. *Journal of Ethnopharmacology*.

[8] Dinan T. G., Cryan J. F. (2017). The microbiome-gut-brain axis in health and disease. *Gastroenterology Clinics of North America*.

[9] Tang R., Wei Y., Li Y. (2018). Gut microbial profile is altered in primary biliary cholangitis and partially restored after UDCA therapy. *Gut*.

[10] Kuczynski J., Stombaugh J., Walters W. A., González A., Caporaso J. G., Knight R. (2011). Using QIIME to analyze 16S rRNA gene sequences from microbial communities. *Current Protocols in Bioinformatics*.

[11] Navas-Molina J. A., Peralta-Sánchez J. M., González A. (2013). Advancing our understanding of the human microbiome using QIIME. *Methods in Enzymology*.

[12] Nakamura T., Yamada K. D., Tomii K., Katoh K. (2018). Parallelization of MAFFT for large-scale multiple sequence alignments. *Bioinformatics*.

[13] Langille M. G., Zaneveld J., Caporaso J. G. (2013). Predictive functional profiling of microbial communities using 16S rRNA marker gene sequences. *Nature Biotechnology*.

[14] Segata N., Izard J., Waldron L. (2011). Metagenomic biomarker discovery and explanation. *Genome Biology*.

[15] Lydersen S., Fagerland M. W., Laake P. (2019). Alternativer til Fishers eksakte test. *Tidsskrift for den Norske Lægeforening*.

[16] Fan C., Zhang D. (2012). A note on power and sample size calculations for the Kruskal-Wallis test for ordered categorical data. *Journal of Biopharmaceutical Statistics*.

[17] Spychala M. S., Venna V. R., Jandzinski M. (2018). Age-related changes in the gut microbiota influence systemic inflammation and stroke outcome. *Annals of Neurology*.

[18] Liang S., Wu X., Jin F. (2018). Gut-brain psychology: rethinking psychology from the microbiota-gut-brain axis. *Frontiers in Integrative Neuroscience*.

[19] Zhao L., Xiong Q., Stary C. M. (2018). Bidirectional gut-brain-microbiota axis as a potential link between inflammatory bowel disease and ischemic stroke. *Journal of Neuroinflammation*.

[20] Hug A., Dalpke A., Wieczorek N. (2009). Infarct volume is a major determiner of post-stroke immune cell function and susceptibility to infection. *Stroke*.

[21] Klehmet J., Harms H., Richter M. (2009). Stroke-induced immunodepression and post-stroke infections: lessons from the preventive antibacterial therapy in stroke trial. *Neuroscience*.

[22] Vogelgesang A., Grunwald U., Langner S.¨. (2008). Analysis of lymphocyte subsets in patients with stroke and their influence on infection after stroke. *Stroke*.

[23] Tascilar N., Irkorucu O., Tascilar O. (2010). Bacterial translocation in experimental stroke: what happens to the gut barrier?. *Bratislavské Lekárske Listy*.

[24] Caso J. R., Hurtado O., Pereira M. P. (2009). Colonic bacterial translocation as a possible factor in stress-worsening experimental stroke outcome. *American Journal of Physiology. Regulatory, Integrative and Comparative Physiology*.

[25] Winek K., Meisel A., Dirnagl U. (2016). Gut microbiota impact on stroke outcome: fad or fact?. *Journal of Cerebral Blood Flow and Metabolism*.

[26] Yamashiro K., Tanaka R., Urabe T. (2017). Gut dysbiosis is associated with metabolism and systemic inflammation in patients with ischemic stroke. *PLoS One*.

[27] Zeng X., Gao X., Peng Y. (2019). Higher risk of stroke is correlated with increased opportunistic pathogen load and reduced levels of butyrate-producing bacteria in the gut. *Frontiers in Cellular and Infection Microbiology*.

[28] Chang X., Feng J., Guo X., Huang M., Nie G., Zhang J. (2018). Dietary supplementation withRehmannia glutinosaaffects the composition of intestinal microorganisms in common carp. *Journal of Basic Microbiology*.

[29] Chen R., Xu Y., Wu P. (2019). Transplantation of fecal microbiota rich in short chain fatty acids and butyric acid treat cerebral ischemic stroke by regulating gut microbiota. *Pharmacological Research*.

